This article has been retracted.

# Clinico-demographic and survival profile of people living with HIV on antiretroviral treatment

**DOI:** 10.3389/fpubh.2023.1084210

**Published:** 2023-03-30

**Authors:** Riyaz Ahamed Shaik, Sharan K. Holyachi, Mohammad S. Ahmad, Mohammed Miraj, Mansour Alzahrani, Ritu Kumar Ahmad, Bader A. Almehmadi, Mohammed Zaid Aljulifi, Meshari A. Alzahrani, Mashael B. Alharbi, Mohammed Muzammil Ahmed

**Affiliations:** ^1^Department of Family and Community Medicine, College of Medicine, Majmaah University, Al Majma'ah, Saudi Arabia; ^2^Department of Community Medicine, Koppal Institute of Medical Sciences, Koppal, Karnataka, India; ^3^Department of Physical Therapy and Health Rehabilitation, College of Applied Medical Sciences, Majmaah University, Al Majma'ah, Saudi Arabia; ^4^Department of Physiotherapy, College of Applied Medical Science, Buraydah Private Colleges, Buraydah, Saudi Arabia; ^5^Department of Medicine, College of Medicine, Majmaah University, Al Majma'ah, Saudi Arabia; ^6^Department of Urology, College of Medicine, Majmaah University, Al Majma'ah, Saudi Arabia; ^7^Ministry of Health, Riyadh, Saudi Arabia; ^8^Department of Basic Medical Sciences, College of Medicine, Majmaah University, Al Majma'ah, Saudi Arabia

**Keywords:** HIV, CD4 counts, tuberculosis, risk factors, ART, retroviral agents

## Abstract

**Objective:**

To assess the demographic, clinical, and survival profile of people living with HIV.

**Methods:**

A retrospective cohort study was conducted among patients enrolled at a single antiretroviral therapy center in North Karnataka. A total of 11,099 were recruited from April 2007 to January 2020, out of which 3,676 were excluded and the final 7,423 entries were subjected to analysis. The outcome of interest was the time to death in months of people living with HIV on antiretroviral therapy (ART). The clinical and demographic characteristics were examined as potential risk factors for survival analysis. To investigate the factors that influence the mortality of patients using ART, univariate and multivariate Cox regression were performed. Hazard ratio (HR), 95% confidence interval (CI), and *p*-values were presented to show the significance. The log-rank test was used to determine the significance of the Kaplan–Meier survival curve.

**Results:**

Out of 7,423 HIV-positive people, majority were female (51.4%), heterosexual typology (89.2%), and in the age group 31–45 years (45.5%). The risk of death in male patients was 1.24 times higher (95% CI: 1.14–1.35) than female patients. Patients with age >45 were 1.67 times more likely to die than patients ≤30 (95% CI: 1.50–1.91). In the multivariable analysis, the hazards of mortality increased by 3.11 times (95% CI: 2.09–2.79) in patients with baseline CD4 count ≤50 as compared to those who had baseline CD4 count >200. The risk of death in patients who were diagnosed with TB was 1.30 times more (95% CI: 1.19–1.42) than in those who did not have TB. The survival probabilities at 3 and 90 months were more in female patients (93%, 70%) compared with male patients (89, 54%), respectively.

**Conclusion:**

This study proved that age, sex, baseline CD4 count, and tuberculosis (TB) status act as risk factors for mortality among people with HIV. Prevention strategies, control measures, and program planning should be done based on the sociodemographic determinants of mortality.

## Introduction

As per 2020 UNAIDS fact sheet (1), 38 million people are living with human immunodeficiency virus (HIV) globally. In 2019, a total of 1.7 million newly infected cases of HIV have occurred, and 690,000 people died of acquired immunodeficiency syndrome (AIDS)-related illnesses globally. Globally, 2.6 million people have access to ART regimens, and 67% of the diagnosed HIV population were accessing ART. The reported HIV prevalence in India among adult male patients was 0.24 and 0.20% among adult female patients, as per National AIDS Control Organization (NACO) report. In 2019, there were 69.22 thousand new infections, 23.48 lakh people are living with HIV, and an estimated 58.96 thousand AIDS-related deaths (2). The primary mode of transmission of HIV among adults is insecure heterosexual intercourse. Another significant mode is mother-to-child transmission, which can occur in utero during pregnancy and intrapartum during labor and delivery (3, 4). Combined antiretroviral therapy is one of the most successful public health interventions in recent times, with increased survival, and individual and societal improvement. The success has been possible because of the simplicity of use, its potency, and its low side effect profile (5). HIV infection being a long-term chronic disease causes morbidity and mortality. Long-term comorbidities and adverse effects can occur due to the disease or the treatment *per se*. In this context, accurate data on the causes of death are of great importance and should help to define priorities in the prevention and management of lethal comorbidities. Such evidence has come from previous prospective studies on people with HIV (6–8). These kinds of studies are not available for the Indian subpopulation, and there is a gap in the understanding of factors affecting the long-term mortality among patients with HIV-positive in India. Although efforts have been made in reducing mortality and extending the life expectancy in people living with HIV (PLHIV), there is considerable morbidity and mortality caused by the disease.

On 1 April 2004, the Government of India launched free ART program for the benefit of all people with HIV. Since then, enrollment and access to ART have improved. AIDS not only remains a serious public health issue but also has a grave impact on the socioeconomic development of the nation. This is attributed to the disease occurrence in the young adult working population, which is the economically productive age group (15–44 years) (2). In 2015, the World Health Organization (WHO) reported that 11% of the 10.4 million new cases of TB infection globally occurred in HIV-positive individuals (9). TB was the leading cause of mortality among people with HIV, and nearly 300,000 people died from HIV-associated TB in 2017 (10). Both TB and HIV significantly affect the human immune system by their ability to evade immune surveillance and clearance, although the mechanism is not fully understood (11). As compared with the general population, the risk of latent TB activation increases 20-fold in people with HIV (12).

There are few studies on mortality at an early stage among PLHIV soon after the initiation of ART which is unlikely to be caused due to drug efficacy (13–15). This indicates that there are several other factors that can indirectly contribute to mortality among people living with HIV, which are often poorly understood (16). Identification and rectification of these modifiable factors during routine clinical care might help in prolonging survival, thereby preventing more deaths among PLHIV. In the Indian context, few retrospective studies with large sample sizes have been conducted to calculate the mortality risks for PLHIV (17, 18). The mortality risk was higher in PLHIV with a baseline CD4 count of <200 (HR: 1.83, 95% CI: 1.47, 2.27), and it was considerably higher in those 50 years or older at the time of registration (HR: 3.01, 95% CI: 2.37, 3.83). In India, only one such retrospective study from 2006 to 2011 was carried out to evaluating the integrated Samastha HIV-prevention cum care and support program in Karnataka (18). Hence, this study was planned to fill in these lacunae by studying a wide population of PLHIV and studying the age, gender, CD4 count, and coexisting tuberculosis infection influence on the long-term mortality of PLHIV.

## Methods

### Study design and population

A retrospective descriptive cohort study was conducted in a single antiretroviral therapy (ART) center, District hospital, Koppal, India, which is the largest and single facility in the district providing screening and treatment facilities for people living with HIV. The study population was the people with HIV receiving ART from the study setting. The study was conducted from April 2007 to January 2020. The data retrieved were regarding the age, gender, HIV diagnosis, treatment status, lab parameters, tuberculosis co-infection, and survival status.

### Procedures

A total of 11,099 patients enrolled in the ART center from different districts of North Karnataka were included in the study. Standard ART and anti-TB therapy registries, electronic formats, patient medical records (cards), and intake forms were used as data sources. Five nurses with training and experience working in the ART and TB clinics at the hospital were involved in the data extraction process. To assure data quality, an experienced supervisor followed up on the extraction processes. Throughout the data extraction process, the researchers and the supervisor continuously checked the checklists for consistency and completeness. A total of 3,676 people were excluded from the study due to the non-availability of complete data, mismatch between the date of registration, death, initiation of ART, and missing values (Figure 1). Data anonymity and confidentiality were maintained throughout the study.

**Figure 1:** Data extraction and validation.

### Statistical analysis

The outcome of interest was the time to death in months among PLHIV on ART. The demographic and clinical variables were analyzed as risk factors for survival analysis. Descriptive statistics were used to present the demographic and clinical characteristics of PLHIV on ART. Both univariate and multivariate Cox regression were used to explore the determinants of mortality of patients on ART. Variables such as sex, age, baseline CD4 count, typology, TB diagnosis, and ART drug regimen were subjected to univariate Cox-regression analysis. Those which were found significant were again subjected to multivariate Cox-regression analysis. Cox regression was first used to obtain risk factors, and then, the survival analysis curves were constructed using these risk factors. Kaplan–Meier survival curve was used to visualize intergroup differences of the risk factors of the survival analysis, and its significance was tested by log-rank test. Survival probabilities were also calculated according to risk factors at different points in time. Hazard ratios (HRs) along with 95% CI and *p*-values are presented to show the significance. *p*-value <0.05 was considered statistically significant. RStudio Version 1.3.1093 was used for statistical analysis (19).

### Ethics approval

The study received ethics approval and waiver of written informed consent from the institutional human ethical committee, Koppal Institute of medical sciences, Koppal, with No. KIMS-Koppal/IEC/53/2020-21.

## Results

A total of 7,423 people living with HIV were included in the analysis. Table 1 presents the demographic and clinical characteristics of the cohort. The majority (45.5%) of the cohort were between 31 and 45 years. The median age of people living with HIV at the start of ART was 35 years with an interquartile range of 27–42 years. The proportion of female patients was higher than male patients (51.4 vs. 48.2%), and 33 (0.4%) were transgender people. Heterosexual typology (89.2%) was the most common sexual orientation. The majority of patients (56.9%) had a CD4 count of >200 mm^3^ and 5.7% had a CD4 count of <50 mm^3^. Only 1,538 (20.7%) patients were diagnosed with TB. Among 1,538 patients with TB, the majority (41.2%) had pulmonary TB (microbiologically confirmed), 40.2% had extrapulmonary TB (clinically diagnosed), and 18.6% had pulmonary tuberculosis (clinically diagnosed). A-TLE was the most common ART regimen used by 62.3% of patients, followed by A-ZLN among 15.8% and A-SLN among 12.8% of patients. The remaining 9.4% of patients were on other miscellaneous ART regimens.

**Table 1:** Demographic and clinical characteristics of patients with HIV on ART (*N* = 7,423).

**Characteristics**	**Number of patients (%)**
**Gender**	
Female	3,813 (51.4%)
Male	3,577 (48.2%)
Transgender people	33 (0.4%)
**Age group**	
≤ 30 years	2,925 (39.4%)
31–45 years	3,378 (45.5%)
>45 years	1,120 (15.1%)
**Baseline CD4 count (mm** ^3^ **)**	
≤ 50	421 (5.7%)
51–200	2,775 (37.4%)
>200	4,227 (56.9%)
**Typology of infection**	
Heterosexual	6,621 (89.2%)
Mother to child	711 (9.6%)
Female sex workers	37 (0.5%)
Men who have sex with men (MSM)	34 (0.5%)
Probable unsafe injection	13 (0.2%)
Blood transfusion	4 (0.1%)
Trucker	2 (0.0%)
Injection drug use (IDU)	1 (0.0%)
**TB diagnosis**	
No	5,885 (79.3%)
Yes	1,538 (20.7%)
**ARV drug regimen** ^*^	
A-TLE	4,621 (62.3%)
A-SLN	931(12.5%)
A-ZLN	1,172 (15.8%)
Others	699 (9.4%)

TG, transgender people ^*^A-TLE, A-SLN, A-ZLN, others.

Out of the 7,423 patients included to receive the ART care, 2,414 (32.5%) died, and 5,009 (67.5%) were censored. The overall median follow-up time for the patients who died was 11 months (IQR 3–30 months), while it was 36 months for the censored patients (IQR 18–61 months). The death rate was high among transgender people (39.4%) followed by male patients (39.0%) and least among female patients (26.4%). In patients with an age of more than 45, the death rate was 42.5%, followed by 36.4% in 31–34 years and 24% in patients aged <30 years. The death rate was noted to be 57.5, 44.9, and 21.9% among patients with a CD4 count of <50, 51–200, and >200 mm^3^, respectively. The death rate among female sex workers (FSWs), men who have sex with men (MSM), and heterosexuals was 40.5, 38.2, and 34.3%, respectively. Death was high among patients with TB (43.2%) as compared to patients without TB (29.7%). The mortality rate was high (73.3%) in the initial 3 months after the start of ART, and it was 63.4, 41.3, and 15.5% at 4–6 months, 7 months−1 year, and >5 years, respectively (Table 2).

**Table 2:** Comparison of demographic and clinical characteristics according to deaths and censored patients.

**Characteristics**	**Number of deaths (%)**	**Number of censored patients (%)**
**Sex**		
Female	1,005 (26.4%)	2,808 (73.6%)
Male	1,396 (39.0%)	2,181 (61.0%)
TS/TG	13 (39.4%)	20 (60.6%)
**Age group**		
≤ 30	704 (24.1%)	2,221 (75.9%)
31–45	1,231 (36.4%)	2,147 (63.6%)
>45	479 (42.8%)	641 (57.2%)
**Baseline CD4 count**		
≤ 50	242 (57.5%)	179 (42.5%)
51–200	1,246 (44.9%)	1,529 (55.1%)
>200	926 (21.9%)	3,301 (78.1%)
**Typology**		
Blood transfusion	1 (25.0%)	3 (75.0%)
FSW	15 (40.5%)	22 (59.5%)
Heterosexual	2,268 (34.3%)	4,353 (65.7%)
IDU	0 (0.0%)	1 (100.0%)
Mother to child	117 (16.5%)	594 (83.5%)
MSM	13 (38.2%)	21 (61.8%)
Probable unsafe injection	0 (0.0%)	13 (100.0%)
Trucker	0 (0.0%)	2 (100.0%)
**TB diagnosis**		
No	1,750 (29.7%)	4,135 (70.3%)
Yes	664 (43.2%)	874 (56.8%)
**Time from start of ART to death/censoring**		
0–3 months	632 (73.3%)	230 (26.7%)
4–6 months	348 (63.4%)	201 (36.6%)
7 months−1 year	335 (41.3%)	477 (58.7%)
1–2 years	378 (32.2%)	797 (67.8%)
2–5 years	489 (19.4%)	2,038 (80.6%)
>5 years	232 (15.5%)	1,266 (84.5%)
**Total**	**2,414 (32.5%)**	**5,009 (67.5%)**
**ART regimen**		
A-TLE	1,106 (23.9%)	3,515 (76.1%)
A-SLN	825 (88.6%)	106 (11.4%)
A-ZLN	325 (27.7%)	847 (72.3%)
Others	158 (22.6%)	541 (77.4%)
**Overall**	**2,414 (32.5%)**	**5,009 (67.5%)**

Bold letters of ‘overall' and ‘total' denotes the PLHIV expereicing death and censoring from time of starting ART.

Table 3 shows the hazard ratios from the univariate and multivariate analyses of the association between the possible determinants of mortality and risk of death. In both univariate and multivariate analyses, sex, age, CD4 count, active TB during treatment, and type of ART regimen showed a statistically significant relationship with mortality (*p*-value < 0.05). It is observed in a multivariate analysis that the risk of death increased 2.41 times more (95% CI: 2.09–2.79) in patients with baseline CD count ≤50 mm^3^ as compared to those who had CD count >200 mm^3^. The risk of death in male patients was 1.24 times higher (95% CI: 1.14–1.35) as compared to female patients. Patients with age >45 were 1.67 times more likely to die (95% CI: 1.50–1.91) than those ≤30 years, and people between 31 and 40 years were 1.28 times more likely to die (95% CI: 1.16–1.41). The risk of death in patients who were diagnosed with TB was 1.30 times more (95% CI: 1.19–1.42) than in those without TB. Mortality was considerably less with A-TLE (adjusted HR 0.13, 95% CI: 0.12–0.14), A-ZLN (adjusted HR 0.13, 95% CI: 0.12–0.15), and other ART (adjusted HR 0.14, 95% CI: 0.12–0.17) regimens, as compared to A-SLN.

**Table 3:** Cox regression model to explore determinants of mortality [hazard ratio (HR) of mortality of patients on ART].

**Determinants**	**Univariate analysis**		**Multivariate analysis**	
	**HR (95% CI)**	***p*** **-value**	**HR (95% CI)**	***p*** **-value**
**Sex**				
Female (Ref)	1		1	
Male	1.64 (1.52–1.78)	< 0.001	1.24 (1.14–1.35)	< 0.001
TS/TG	1.76 (1.02–3.04)	0.044	1.47 (0.85–2.54)	0.172
**Age groups (in years)**				
≤ 30 (Ref)	1		1	
31–45	1.61 (1.47–1.77)	< 0.001	1.28 (1.16–1.41)	< 0.001
>45	2.13 (1.90–2.40)	< 0.001	1.67 (1.48–1.88)	< 0.001
**Baseline CD4 count**				
>200 (Ref)	1		1	
≤ 50	3.48 (3.02–4.00)	< 0.001	2.41 (2.09–2.79)	< 0.001
51–200	2.31 (2.12–2.52)	< 0.001	1.69 (1.55–1.84)	< 0.001
**TB diagnosis**				
No (Ref)	1		1	
Yes	1.39 (1.27–1.52)	< 0.001	1.30 (1.19–1.42)	< 0.001
**ART regimen**				
A-SLN (Ref)	1		1	
A-TLE	0.11 (0.10–0.12)	< 0.001	0.13 (0.12–0.14)	< 0.001
A-ZLN	0.11 (0.10–0.13)	< 0.001	0.13 (0.12–0.15)	< 0.001
Others	0.10 (0.08–0.12)	< 0.001	0.14 (0.12–0.17)	< 0.001

Overall median survival time was 90 months with an interquartile range of 86.46–93.45 months. Statistically significant differences (*p*-value <0.001) in median survival times were observed with gender, age group, baseline CD4 count, TB status, and ART regimen. As compared to male patients (71, IQR: 65.83, 76.17), the median survival time in months was higher among female patients (99, IQR; 97.49–101.51, *p*-value < 0.001) and transgender population (66, IQR: 5.53–1,126.47, *p* = 0.043). With regard to the age group, the median survival time decreased with increasing age, while the median survival time increased in patients with a baseline CD4 count of >200 mm^3^. As compared to people without TB (98.00, IQR 95.83–100.18), people with TB had lower median survival time (69, IQR; 62.23–75.77, *p* < 0.01). As compared to people on the A-TLE regimen (96, IQR: 92.37–99.63), people on A-SLN had significantly median lower survival time (6, IQR: 5.17–6.83, *p* < 0.01). In comparison, people with A-ZLN (101, IQR could not be computed, *p* < 0.01) and other regimens (99, IQR: 95.67–102.33, *p* < 0.01) had higher median survival time (Table 4).

**Table 4:** Comparison of median survival times across various explanatory parameters.

**Parameter**	**Median**				**Log rank test (*p*-value)**
	**Estimate**	**SE**	**95% CI**		
			**LB**	**UB**	
**Gender**					
Male	71.00	2.64	65.83	76.17	
Female	99.00	0.77	97.49	100.51	< 0.001
TS/TG	66.00	30.85	5.53	126.47	0.043
**Age group**					
≤ 30 years	100.00	1.24	97.57	102.43	< 0.001
31–45 years	82.00	2.81	76.50	87.50	
>45 years	59.00	5.12	48.96	69.04	
**Baseline CD4 count**					
≤ 50	34.00	6.85	20.58	47.42	< 0.001
51–200	36.00	2.43	31.25	40.75	
>200	101.00	1.23	98.58	103.42	
**Status of TB**					
No	98.00	1.11	95.83	100.18	< 0.001
Yes	69.00	3.46	62.23	75.77	
**ART regimen**					
A-TLE	96.00	1.85	92.37	99.63	
A-SLN	6.00	0.43	5.17	6.83	< 0.001
A-ZLN^*^	101.00				< 0.001
Others	99.00	1.70	95.67	102.33	< 0.001

* Median values could not be computed.

The median survival time of patients in the age group ≤30, 31–45, and >45 years was ~100, 82, and 59 months, respectively. The log-rank test for difference in survival gives a *p*-value < 0.0001, indicating that the age groups differed significantly in survival.

The median survival of patients with baseline CD4 count ≤50, 51–200, and >200 mm^3^ was ~26, 60, and 101 months, respectively. The log-rank test for difference in survival gives a *p*-value < 0.0001, indicating that there was a significant difference in survival pattern observed in patients with different baseline CD4 counts (Table 5 and Figure 2).

**Table 5:** Survival probabilities according to risk factors at a different point in time.

**Characteristics**		**Time in months**				
		**3**	**6**	**12**	**24**	**60**
Sex	Male	89%	84%	78%	70%	54%
	Female	93%	89%	85%	80%	70%
	TS/TG	87%	81%	77%	65%	43%
Age group	≤ 30 years	94%	91%	87%	83%	72%
	31–45 years	90%	85%	79%	72%	59%
	>45 years	87%	79%	74%	65%	49%
Baseline CD4	≤ 50	77%	68%	61%	52%	38%
	51–200	86%	80%	72%	65%	50%
	>200	96%	93%	90%	85%	74%
TB diagnosis	No	92%	87%	82%	77%	65%
	Yes	91%	85%	79%	70%	54%
ART regimen	A-TLE	95%	93%	90%	85%	71%
	A-SLN	66%	49%	32%	15%	4%
	A-ZLN	93%	89%	84%	79%	71%
	Others	95%	93%	90%	84%	74%

**Figure 2:** Kaplan-Meier Survival curves showing intergroup differences with respect to **(A)** Sex, **(B)** Age, **(C)** CD4 Count, **(D)** Tuberculosis (TB), and **(E)** ART Regimen.

## Discussion

This retrospective descriptive cohort study was conducted considering the data of patients from April 2007 to January 2020. The findings of this study showed that the most commonly affected age group was 31–45 years, and female patients were most commonly affected. The heterosexual route was the commonest mode of transmission among study participants. Sex, age group, baseline CD4 count, and TB diagnosis have a significant relationship with the mortality of patients with HIV-positive.

Among the study population, 51.4% were female patients. The most commonly affected age group was 31–45 years. These findings were similar to the study by Kumawat et al. (20), where the most commonly affected age group was 15–49 years, and in contrast to the current study, male patients were most commonly affected. This difference may be due to the low sample size of 300 in their study, hence, reducing the representativeness of the HIV-positive population. The observation of female patients becoming infected with HIV is consistent with the global HIV/AIDS trend, which shows that the epidemic is affecting more women than men, and the number of women living with the virus outnumbers men by a large margin (21, 22).

Transmission through heterosexual contact was most common (89.2%) among the study participants, followed by mother-to-child transmission. Similar findings were observed in previous studies by Kumawat et al. (20) (87.67%), Joge et al. (23) (94.39%), and Jha et al. (24) (72.2%).

Among the study participants, 20.7% had tuberculosis. A previous study has shown that 10.66% of the 300 participants had tuberculosis (23). Superadded TB infection is one of the most common reasons for mortality in people living with patients with HIV, accounting for 26% of AIDS-related deaths and majority (99%) of which occurred in developing countries (11, 25–28). Co-infection control strategies have been developed through early diagnosis of both diseases and adequate, timely treatment (29). According to a 2015 report, the risk of a person with HIV/AIDS developing active TB is 26 times higher compared to the general population (30).

Sex, age group, baseline CD4 count, and TB diagnosis showed a statistically significant relationship with mortality in people with HIV. Our study's finding that male patients have a 1.24 times higher risk of death (95% CI: 1.14–1.35) than female patients builds on previous studies that has shown that men with HIV have a higher risk of death. The findings we present are also consistent with broader health and survival disparities experienced by men around the world at all ages (30, 31).

Mortality was noted to be higher in people with HIV who were more than 45 years (42.8%) compared to ≤30 years (24.1%) and 1.67 times (CI 1.48–1.88) higher and older age group. The age-specific deaths observed in our study are consistent with other studies that found higher mortality in patients aged >50 or 55 years compared to patients aged <50 or 55 years, respectively, with longer follow-up (32, 33). A study done by Mutevedzi et al. (34) reported a higher probability of death among older individuals (>50 years) than younger patients (<50 years) in the first 12 months of ART therapy initiation, but no significant difference in mortality later, suggesting age-related non-HIV causes are the major cause of death among older individuals.

It was observed in the multivariable analysis that hazards of mortality increased by 3.11 times (95% CI: 1.19–1.44) and 2.11 times (95% CI: 1.94–2.30) in patients with baseline CD4 count ≤50 and baseline CD4 count 51–200, respectively, as compared to those who had baseline CD4 count >200. A similar retrospective cohort study done in Oromia region, Ethiopia, on a large population of 2,775 individuals with HIV reported lower mortality (AHR = 0.719; 95% CI: 0.536–0.966) among individuals with CD4 count compared to people living with HIV with CD4 count more than 200 cells/mm^3^ (35). Several studies have found a significant relationship between CD4 cell count and survival rates, implying that a low CD4 cell count is associated with an increased risk of mortality (36–38). Suppression of viral load plays an important role in delaying the progression of the disease and mortality. To achieve viral suppression, routine HIV viral load (VL) monitoring is recommended by the World Health Organization (WHO) (39). This is due to the fact that a decrease in CD4 count, which is a marker of immunological failure, occurs as a result of viral replication, which can, thus, be considered an endpoint (40).

The overall survival probabilities among people with HIV declined over follow-up time with regard to various risk factors such as age, sex, CD4 count, and TB status (Table 5). The survival probabilities at 3 and 90 months were more in female patients (93, 70%) compared with male patients (89, 54%), respectively. This trend was in concordance with Zhang et al. (41) study, and it is due to fact that the ART adherence was higher in female patients who stayed at home and were easily accessible when compared to male patients who did not receive timely interventions and treatment for opportunistic infections.

The survival probability of people with HIV receiving different ART regimens declined over time from 95% at 3 months to 71% at 90 months with the A-TLE regimen. A retrospective cohort study done in China reported the cumulative survival rate at 1, 2, 3, 4, and 5 years, of 97.1, 93.4, 90.6, 88.8, and 86.0%, respectively (41). A similar survival analysis of patients with HIV-positive during the year 1996 to 2013 was done by ART cohort collaboration. The study concluded that in the late ART era, survival during the first 3 years of ART initiation improved, which can be attributed to the transition to less toxic antiretroviral drugs in the early 2000s (42).

Various similar research studies were carried out in the African region (33–39), but the current study is the first of its kind to be carried out in North Karnataka, India. The strength of this current study is that it was done on a relatively large sample size; long-term survival analysis was done. The limitation is that it is a single-center, retrospective study. Prospective, multi-centric studies involving a large population are recommended in future.

## Conclusion

The median survival time was higher in female patients in the age group ≤30 years, patients with baseline CD4 count >200, and patients who were not diagnosed with TB. Tuberculosis was found to be one of the risk factors for mortality in people with HIV. This study has created evidence on the role of age, sex, baseline CD4 count, and TB status as risk factors for deaths among HIV-positive individuals. The finding of survival probabilities with different treatment regimens is the first of its kind for Karnataka state that can help Karnataka State AIDS Prevention and Control Society (KSAPS) to make policy changes with regard to treatment regimens. The National AIDS Control Organization must, therefore, work to create a cutting-edge health system that will give ART at higher CD4 cell count thresholds and put an emphasis on early discovery, testing, sustainable treatment, and enhanced retention.

## Data availability statement

The original contributions presented in the study are included in the article/supplementary material, further inquiries can be directed to the corresponding author.

## Ethics statement

The ethical review committee of the Koppal Institute of Medical Sciences had approved the study experiment (data collection) which was in accordance with institutional ethical guidelines in the purview of the declaration of Helsinki.

## Author contributions

RAS has conceptualized the study and played primary role in compiling, analysis, and interpretation of the data. RAS, MSA, SKH, and MM did the manuscript preparation. BAA and MZA did the manuscript editing. MSA, SKH, and MM approved the final draft. RKA, MBA, and MMA did the data cleaning and data analysis. BAA, RAS, MA, and MAA have contributed in fine tuning of the proposal, manuscript write up, editing, and review. All the authors take complete responsibility for the content of the manuscript, read, and approved final version of the manuscript.
